# Screening Potential Drugs for the Development of NAFLD Based on Drug Perturbation Gene Set

**DOI:** 10.1155/2022/7606716

**Published:** 2022-04-16

**Authors:** Zhengzheng Gao, Lina Dai, Haifeng Zhang

**Affiliations:** Basic Medical College of Inner Mongolia Medical University, Hohhot, China

## Abstract

Nonalcoholic fatty liver disease (NAFLD) has become one of the problems affecting the health of the population worldwide. The progressive disease includes nonalcoholic steatohepatitis (NASH) and fibrosis, which with no approved therapy, system identification of effective drugs remains challenging. In this work, we applicated drug perturbation gene set enrichment analysis to screen drugs for the development of NAFLD. A total 15490 small-molecule compounds were analyzed in our study; based on the *p* value of enrichment score, 7 small-molecule compounds were found to have a potential role in NASH and fibrosis. After pathway analyses, we found indoximod had effects on nonalcoholic fatty liver disease through regulated TNFa, AP-1, AKT, PI3K, etc. Furthermore, we established the NAFLD cell model with LO2 cells induced using PA; ELISA showed that the levels of TG, ALT, and AST were significantly improved by indoximod. In summary, our study offers optimal therapeutic drugs, which may provide novel insight into the precise treatment of NAFLD and promote researches.

## 1. Introduction

Nonalcoholic fatty liver disease (NAFLD) is a common multifactorial liver disease that becomes a common public health problem seriously affecting people's lives and health [1]. NAFLD was considered as a manifestation of the metabolic syndrome which is induced by abnormal deposition of lipid in hepatocytes [2]. Some studies have suggested that NAFLD is strongly associated with hypertension, hyperlipidemia diabetes, and atherosclerosis [3]. Statistics has rapidly implicated the trend rate of growth towards a younger onset becoming a serious medical social problem during recent decades [4]. Therefore, more precise and effective therapeutic strategies for NAFLD are urgently needed.

The pathogenesis of NASH was very complicated. After NASH was defined as a new disease in 1980, Powell et al. found that obesity and diabetes were the main risk factors, and NASH might be a metabolic-related disease [5]. Animal studies have shown that high-fat food or knockout of the thin element receptor induced fatty liver, and fatty liver cells were more sensitive to the damage of inflammatory factors and lipid oxides [6]. Based on these studies, Day and James of the British Liver Research Center proposed the “second strike” theory of the pathogenesis of NASH in 1998 [7], which suggested that fat accumulation and degeneration were the first strike and exposure to inflammatory factors and metabolic by-products were the second strike eventually leading to cell death, inflammation, and fibrosis. With the deepening of clinical and basic research, people have found that the hypothesis of “second strike” was too simplistic. NASH is actually the result of interacting in parallel of multiple risk factors including multiple cell types and multiple tissues and organs, which is the so-called “multiple parallel strikes” theory [8]. The risk factors include insulin resistance, oxidative stress, hormone imbalance, chronic inflammation, fibrosis, immune and intestinal bacterial disorders, and the other various cells in the liver, intestines, and adipose tissue.

NAFLD was contributed by multiple factors in long-term cooperation [9]. Monotherapy for NAFLD is hard to obtain a great therapeutic effect [10]. With the deepening understanding on NAFLD, the therapeutic schedule is becoming more and more diverse [11]. Currently available treatment of NAFLD is divided into three categories: antioxidants, antiobesity pills, and insulin sensitizers [12]. Research has shown that oxidative stress response (OS) was the most important factor in the transformation of NAFLD to NASH. Antioxidant can protect against NAFLD and thereby retard the progress of NAFLD [13]. Kenny et al.'s [14] study reflects that too much lipid accumulated is one of the reasons of NAFLD. Antiobesity pills can facilitate fat metabolism so that it can improve fat metabolism, such as orlistat and sibutramine. Due to the insulin resistance in nonalcoholic fatty liver disease, insulin sensitizers can be used to treat the disease by promoting the binding of insulin to its receptor and accelerating the uptake of glucose into peripheral tissues [15]. However, the clinical manifestations of nonalcoholic fatty liver disease are not only reflected in the hepatobiliary system but also cause dysfunction and changes in other systems [16]. At present, none of the drugs can be absolutely treated, and further research is needed.

In order to screen the potential therapeutic drugs for liver diseases, in the present test, we firstly get the disease high-throughput molecular profiles from the Gene Expression Omnibus (GEO) database, then analyzed the biological functions and pathways of differentially expressed genes, and used drug perturbation gene set enrichment analysis to screen the potential therapeutic drug. Our research will provide strategies for the treatment of NAFLD.

## 2. Materials and Methods

### 2.1. Data Collection and Identification of Differentially Expressed Genes

We get the expression profiling of liver biopsies from the course of nonalcoholic fatty liver disease from the GEO (Gene Expression Omnibus https://www.ncbi.nlm.nih.gov/geo/) database (GSE130970), including 5 normal, 23 nonalcoholic steatohepatitis, and 25 hepatic fibrosis. *T*-test (*p* value < 0.05) was set as the cutoff criteria to evaluate differentially expressed genes (DEGs). The heat maps were plotted based on the pheatmap package of R.

### 2.2. Drug Structure and Drug Expression Profile Data

PubChem (https://pubchem.ncbi.nlm.nih.gov/) is a public repository for archiving biological tests of small molecules generated through high-throughput screening experiments, medicinal chemistry studies, chemical biology research, and drug discovery programs. The drug expression profile data is from the Library of Integrated Network-Based Cellular Signatures (LINCS) L1000 dataset that measured changes in genes before and after treatment of human cells with over 20000 small-molecule compounds including most of the FDA-approved drugs.

### 2.3. Functional Enrichment Analysis

Gene Ontology (GO) annotation and Kyoto Encyclopedia of Genes and Genomes (KEGG) pathway of the DEGs were analyzed and visualized by clusterProfiler package of R. *p* < 0.05 was considered as a threshold of GO and KEGG enrichment analysis.

### 2.4. Drug Perturbation Gene Set Enrichment Analysis (dpGSEA)

dpGSEA is an approach for drug screening, which used the drug perturbation gene set as a background and disease-related characteristic genes for enrichment analysis. In this way, drugs related to characteristic polar shadows can be detected or potential treatments can be discovered [17].

### 2.5. Cell Culture and Treatment

Based on the previous methods of established cellular model of NAFLD [18], normal human hepatocyte cell lines (L02 cells) were used in our study obtained from the Shanghai Institute of Cell Bank. Cells were cultured in DMEM/L media containing 10% fetal bovine serum and 1% penicillin/streptomycin at 37°C with 5% CO_2_. Palmitic acid (PA) was added at a 0.3 mmol/liter concentration for 24 h to establish a cellular model of NAFLD. Cells were divided into control, PA, and PA+indoximod groups. Indoximod (200 *μ*M) was added to cell cultures for 12 h, followed by coincubation with PA for another 24 h. Levels of TG, alanine aminotransferase (ALT), and aspartate aminotransferase (AST) were measured by commercial kits according to the manufacturers' instructions. ELISA kits for TG (SBJ-H0240), ALT (SBJ-H0658), and AST (SBJ-H0027) were purchased from Nanjing Sen Bei Jia Biotechnology (Nanjing, China).

## 3. Results

### 3.1. DEG Analysis for the Course of NAFLD

Firstly, we identified DEGs in different stages of nonalcoholic fatty liver. As shown in Figures 1(a) and 1(b), there were 2894 differentially expressed genes in NASH and 4372 in liver fibrosis. Through the comparison of DEGs between NASH and fibrosis, we found 859 unique DEGs in NASH and 2327 DEGs unique in fibrosis; 2045 differential genes belong to the common (Figure 1(c)).

### 3.2. DEG Functional Enrichment Analysis

Next, we performed GO and KEGG analysis of DEGs. The results had shown that DEGs in NASH are mainly involved in metabolism-related processes, such as purine-containing compound metabolic process, glycerophospholipid metabolic process, and glucose metabolic process which is related to liver function. KEGG analysis results had shown that DEGs mainly participate in regulation of the chemokine signaling pathway and FoxO signaling pathway (Figure 2). Meanwhile, we found small-molecule catabolic process, purine-containing compound metabolic process, herpes simplex virus 1 infection pathway, and chemokine signaling pathway were regulated by DEGs in fibrosis (Figure 3). Furthermore, the chemokine signaling pathway was found to be included in both pathological states. The results showed that inflammatory response plays a key role in the progression of NAFLD.

### 3.3. Drug Screening for the Course of NAFLD

In order to screen potential therapeutic drugs for NAFLD progression, the DEGs in different pathological states of NAFLD as characteristic genes were analyzed by dpGSEA. According to the *p* value of enrichment score (*p* < 0.05), we have individually identified candidate drugs for each pathological state. Finally, we found 7 drugs (or compound) have potential therapeutic effects on NASH and fibrosis (Figure 4): acifran [19], sirolimus, progesterone [20], abexinostat [21], indoximod [22], rutin [23], and bisindolylmaleimide [24]. Furthermore, we performed KEGG analysis on seven candidate drugs based on perturbation gene set. The results had shown that indoximod had effects on nonalcoholic fatty liver disease (Figure 5). We expanded the structure of the pathway. As shown in Figure 6, indoximod influenced the pathological process of nonalcoholic fatty liver disease through regulated TNFa, AP-1, AKT, PI3K, etc. The results indicated that indoximod may be an effective drug for nonalcoholic fatty liver.

### 3.4. Indoximod Alleviated PA-Induced Lipid Accumulation and Hepatocyte Injury

We further confirmed the potential role of indoximod through cell experiments; we used PA treatment hepatocytes to establish the NAFLD cell model. The pathological alterations of livers were evaluated by the content of triglyceride and the levels of circulating for liver enzyme. PA induced lipid accumulation and hepatocyte injury consistent with previous studies [25, 26], which were manifested by the increasing levels of TG, ALT, and AST. As indoximod was applied, triglyceride accumulation and liver injury were significantly reduced (Figures 7(a)–7(c)). The results had showed that indoximod had the potential to treat NAFLD.

## 4. Discussion

NAFLD is the most difficult to treat in the field of metabolic diseases. Although a great deal of studies on pathogenesis of NASH have made a great many of progress over these years, there have been no drugs approved so far [27]. With the popularity of Chinese metabolic diseases including obesity and diabetes, the pressure of NASH in the future cannot be underestimated [28, 29].

After years of research, our understanding of the pathogenesis of NASH has made great progress, but I think there is still a long way to go before finding an effective treatment for NASH [30]. From the above incomplete combing of NASH targets, it can be seen that the current targets for NASH are not too few but too many, and no real effective targets have been found [31]. The current research is only for the known signal pathways and the ways and technical means that can be intervened. The development of multiple omics technology, genetics, proteomics, genomics, and metabolomics will help us have a better understanding of the development of NAFLD [32].

In this research, we integrated the disease high-throughput molecular profiles and drug perturbation profiles and then considered directionality of gene modulation of drug.

We successfully identified seven drugs that have a potential role in HASH and fibrosis, including acifran, sirolimus, progesterone, abexinostat, indoximod, rutin, and bisindolylmaleimide. Consistent with the results of Hyo-Kyoung Choi's study, they found that rutin and its metabolites as novel histone acetyltransferase (HAT) inhibitors suppress the progression of nonalcoholic fatty liver disease. In addition, the other six drugs were all reported to be related to hepatic disease. Acifran has the effect of lowering blood lipids; sirolimus, bisindolylmaleimide, and abexinostat have been reported to have the effect of treating liver cancer; and progesterone and indoximod have the effect of reducing liver damage. This result also suggested that these six drugs may have potential therapeutic effects on NAFLD. Through the pathway analysis, we found that indoximod could influence nonalcoholic fatty liver. Finally, we verified the effectiveness of indoximod through cell experiments. There are certain limitations to our study. We will investigate the mechanism of indoximod in treatment of NAFLD.

Taken together, our experiment data provided a potential therapeutic agent for the development of NAFLD; meanwhile, it also provided ideas for screening new drugs for complex diseases.

## Figures and Tables

**Figure 1:** Differentially expressed genes in each type of NAFLD. Unsupervised hierarchical clustering analysis is used. The lower and higher expression values are represented by blue and the red colors, respectively. (a) Heat maps show differentially expressed genes in NASH. (b) Heat maps show differentially expressed genes in hepatic fibrosis. (c) Venn plots of differentially expressed genes associated with each type of NAFLD.

**Figure 2:** GO enrichment and enrichment in KEGG pathway analysis of the DEmRNA in NASH: (a) biological process of DEmRNAs; (b) KEGG pathway of DEmRNAs.

**Figure 3:** GO enrichment and enrichment in KEGG pathway analysis of the DEmRNA in hepatic fibrosis: (a) biological process of DEmRNAs; (b) KEGG pathway of DEmRNAs.

**Figure 4:** The common drugs of potential therapeutic effects on NASH and hepatic fibrosis.

**Figure 5:** Enrichment in KEGG pathway analysis of indoximod perturbation gene set.

**Figure 6:** The structure visualization of nonalcoholic fatty liver disease pathway influenced by indoximod.

**Figure 7:** Impact of indoximod on PA-induced production of lipid profile. Measurement of intracellular levels of (a) triglycerides, (b) alanine aminotransferase, and (c) aspartate aminotransferase by ELISA. Data are shown as the mean ± SE. ^∗∗^*p* < 0.01 vs. Con group; ^#^*p* < 0.05 vs. PA group. TG: triglycerides; ALT: alanine aminotransferase; AST: aspartate aminotransferase.

## Data Availability

Previously reported (high-throughput sequencing) data were used to support this study and are available at https://www.ncbi.nlm.nih.gov/geo/query/acc.cgi?acc=GSE130970. These prior studies (and datasets) are cited at relevant places within the text as references [Hoang SA, Oseini A, Feaver RE, Cole BK et al., Gene expression predicts histological severity and reveals distinct molecular profiles of nonalcoholic fatty liver disease, Sci Rep 2019 Aug 29; 9(1): 12541. PMID: 31467298].
